# MicroRNA-200a Inhibits Inflammation and Atherosclerotic Lesion Formation by Disrupting EZH2-Mediated Methylation of STAT3

This article has been retracted.

**DOI:** 10.3389/fimmu.2020.00907

**Published:** 2020-06-23

**Authors:** Jinpeng Wang, Ping Li, Xiaofei Xu, Beilin Zhang, Jing Zhang

**Affiliations:** ^1^Department of Cardiology, The Second Hospital of Jilin University, Changchun, China; ^2^Department of Developmental Pediatrics, The Second Hospital of Jilin University, Changchun, China; ^3^Department of Radiology, The Second Hospital of Jilin University, Changchun, China; ^4^Department of Physiology, College of Basic Medical Sciences, Jilin University, Changchun, China

**Keywords:** atherosclerosis, inflammation, microRNA-200a, EZH2, STAT3

## Abstract

Endothelial inflammation and dysfunction are critical to the process of atherosclerosis. Emerging evidence demonstrates that upregulation of miR-200a reduces VCAM-1 expression and prevents monocytic cell adhesion onto the aortic endothelium. However, limited information is available about the role of microRNA-200a (miR-200a) in facilitating atherosclerotic lesion formation. We investigated the anti-inflammatory and anti-atherosclerotic actions of miR-200a. Human umbilical vein endothelial cells (HUVECs) were cultured in the presence of oxidized low-density lipoprotein (ox-LDL), and their viability and apoptosis were evaluated using CCK-8 assays and flow cytometric analysis. The enhancer of zeste homolog 2 (EZH2) promoter activity was evaluated in the presence of miR-200a by dual luciferase reporter gene assay. EZH2-mediated methylation of signal transducer and activator of transcription 3 (STAT3) was validated by ChIP and IP assays. ApoE^−/−^ mice were given a 12-week high-fat diet and developed as *in vivo* atherosclerotic models. miR-200a was downregulated but EZH2 and HMGB1 were upregulated in ox-LDL-treated HUVECs and the aorta tissues of atherosclerotic mouse models. Elevated miR-200a was shown to protect HUVECs against ox-LDL-induced apoptosis and inflammation. EZH2 was verified as a target of miR-200a. The protective effects of miR-200a were abrogated upon an elevation of EZH2. EZH2 methylated STAT3 and enhanced STAT3 activity by increased tyrosine phosphorylation of STAT3, thereby increasing apoptosis and release of pro-inflammatory cytokines in ox-LDL-treated HUVECs. An anti-atherosclerotic role of miR-200a was also demonstrated in atherosclerotic mouse models. Our study demonstrates that miR-200a has anti-inflammatory and anti-atherosclerotic activities dependent on the EZH2/STAT3 signaling cascade.

## Introduction

Atherosclerosis is a chronic inflammatory disease involving arteries (1). Atherosclerosis, a leading cause of morbidity and mortality, is characterized by the formation of vascular plaques (2). Atherosclerosis is responsible for acute myocardial infarction and cerebrovascular accidents and accounts for the large majority of cardiovascular deaths (3). It has been reported that endothelial dysfunction is central to the progression of atherosclerosis (4). Oxidized low-density lipoprotein (ox-LDL) is demonstrated to participate in the pathogenesis of atherosclerosis by inducing inflammatory responses (5). Although there have been great advancements in new therapeutics for atherosclerosis treatment, significant morbidity from atherosclerosis is prevalent globally (6). Therefore, there exists a significant need to investigate the pathological mechanisms underpinning atherosclerosis and identify novel molecular targets for devising atherosclerosis treatments.

MicroRNAs (miRNAs) are known as small noncoding RNA molecules that regulate gene expression and are implicated in multiple biological processes, including atherosclerosis (7). Abundant evidence has revealed that several miRNAs, including miR-210, are implicated in atherosclerotic plaque formation (8). miR-200a belongs to the miR-200 family, which is regarded as a tumor inhibitor and is reported to be poorly expressed in various human cancers (9). Inflammation is a key pathological process in atherosclerosis, and miR-200a has been reported to modulate endothelial inflammation induced by high glucose by targeting O-linked N-acetylglucosamine transferase (10). However, the molecular mechanism of miR-200a involvement and how it contributes to atherosclerosis remains unclear. Preliminary microarray analysis in the present study has suggested that enhancer of zeste homolog 2 (EZH2) is a target gene of miR-200a. EZH2, as a catalytic subunit of Polycomb repressive complex 2, can trimethylate lysine 27 of histone 3 and epigenetically inhibit transcription of developmentally regulated genes (11). Existing literature has indicated that some miRNAs, such as miR-101 and miR-214, can directly target EZH2 expression, and a role of EZH2 in atherosclerosis has been validated (12). In addition, EZH2 is known to regulate DNA methylation by mediating the activity of DNA methyltransferases (13). EZH2 is verified to bind to and methylate signal transducer and activator of transcription 3 (STAT3), contributing to its activation (14). STAT3 is also implicated in the development of atherosclerosis by regulating cellular processes, such as cell growth and apoptosis (15). Furthermore, STAT3 can affect the high mobility group box 1 protein (HMGB1) expression during inflammatory responses (16). A role of HMGB1 in atherosclerosis progression has also been reported (7). However, the putative role of miR-200a-mediated regulation of EZH2 via the STAT3/HMGB1 axis on atherosclerosis remains unclear. In the present study, the putative role of miR-200a in modulating the inflammatory cascade central to atherosclerosis and its possible mechanisms are explored, which may provide theoretical basis for developing novel directions for treating atherosclerosis.

## Materials and Methods

### Ethics Statement

All animal experiment protocols were approved by the “Ethics Committee of Medical Experiment Animals in the College of Basic Medicine of Jilin University.” Animal experiments were conducted in strict accordance with the “Guide for the Care and Use of Laboratory Animals” published by the US National Institutes of Health. Great efforts were made to minimize the number of animals used in the experiments and their suffering.

### Cell Treatment

The human umbilical vein endothelial cell line, HUVEC, was obtained from American Type Culture Collection (ATCC, Manassas, VA, USA). Cells were cultured in the vascular cell basal medium (Gibco, Rockville, MD, USA) supplemented with 10% fetal bovine serum and antibiotics (100 mg/ml streptomycin and 100 IU/ml penicillin) (Gibco) in an incubator with 5% CO_2_ at 37°C (6). HUVECs at passage 2–4 were used for subsequent experiments (17). The cell models of atherosclerosis were established in a medium containing 0, 20, and 40 μg/ml ox-LDL (Beijing Solarbio Science and Technology Co. Ltd., Beijing, China) for 0, 24, and 48 h, respectively. miR-200a mimic, miR-200a inhibitor, small interfering RNA (siRNA) targeting EZH2, siRNA targeting HMGB1, expression vectors containing EZH2, and HMGB1 (GenePharm Co., Ltd., Suzhou, Jiangsu, China) were transfected into 20 μg/ml ox-LDL-treated HUVECs (24 h) using Lipofectamine 2000 reagent (Invitrogen, Carlsbad, CA, USA). Transient transfection lasted for 48 h. miR-negative control (miR-NC) mimic, miR-NC inhibitor, scramble siRNA, and empty vector served as negative controls (GenePharm).

### Animals and Establishment of Atherosclerosis Model

A total of 36 specific pathogen-free C57BL/6J ApoE^−/−^ male mice (weighing 16–21 g; aged 4–6 weeks old) were fed on a standard chow diet (*n* = 12) or a high-fat diet (0.25% cholesterol, 15% fat) (*n* = 24) (1). A high-fat diet was provided for 12 weeks in order to induce atherosclerosis in ApoE^−/−^ mice (18). miR-200a agomir (Lot No.: 4736, GenePharm) with Invivofectamine 3.0 (Thermo Fisher, MA, USA) was further injected into ApoE^−/−^ mice at 7 mg/kg/day via tail vein to upregulate miR-200a, with NC agomir (agomir-NC, Lot No.: 170601, GenePharm) as NC for 10 days, once a day. After 12 weeks, mice were fasted for 12 h before euthanasia and then euthanized via anesthesia with 3% pentobarbital. Thereafter, three mice in each group were randomly selected for the experiment. Overall, 6 ApoE^−/−^ mice died during the experiment and 30 ApoE^−/−^ mice survived (83.33%), and these were randomly classified into 3 groups, with 10 mice in each group.

### RNA Isolation and Quantitation

Total RNA was extracted from HUVECs using TRIZOL (Invitrogen). Next, total RNA was reversely transcribed into cDNA using the TaqMan™ MicroRNA Reverse Transcription Kit (4366596; Thermo Fisher) and High-Capacity cDNA Reverse Transcription Kit (4368813; Thermo Fisher). Glyceraldehyde-3-phosphate dehydrogenase (GAPDH) and U6 (Invitrogen) were used as internal reference for mRNA and miRNA amplification, respectively. The reverse transcription quantitative polymerase chain reaction (RT-qPCR) was performed using SYBR®Premix Ex TaqTM kit (Tli RNaseH Plus) (RR820A; TaKaRa, Kyoto, Japan) with primers for miR-200a, EZH2, and HMGB1 (designed and synthesized by Invitrogen; Table 1) on the Mx3000p Sequence Detection System (Agilent Technologies, USA). Relative expression levels were determined using the 2^−ΔΔCt^ method.

**Table 1:** Primer sequences for RT-qPCR.

**Target**	**Sequences (5^**′**^-3^**′**^)**
Hsa-miR-200a	F: TTCCACAGCAGCCCCTG
	R: GATGTGCCTCGGTGGTGT
Mum-miR-200a	F: CCTACGCCACAATTAACAAGCC
	R: GCCGTCTAACACTGTCTGGTA
EZH2 (human)	F: AATCAGAGTACATGCGACTGAGA
	R: GCTGTATCCTTCGCTGTTTCC
U6 (human)	F: CTCGCTTCGGCAGCACA
	R: AACGCTTCACGAATTTGCGT
U6 (mouse)	F: GCATGACGTCTGCTTTGGA
	R: CCACAATCATTCTGCCATCA
GAPDH (human)	F: GGAGCGAGATCCCTCCAAAAT
	R: GGCTGTTGTCATACTTCTCATGG

*RT-qPCR, reverse transcription quantitative polymerase chain reaction; miR-200a, microRNA-200a; EZH2, enhancer of zeste homolog 2; GAPDH, glyceraldehyde-3-phosphate dehydrogenase; F, forward; R, reverse*.

### Western Blot Analysis

Total protein was extracted from HUVECs using radio-immunoprecipitation assay cell lysis (R0010; Solarbio) and refined using a bicinchoninic acid protein assay kit (GBCBIO Technologies, Guangzhou, Guangdong, China). The proteins (40 μg) were separated using 10% sodium dodecyl sulfate-polyacrylamide gel electrophoresis and transferred onto the polyvinylidene fluoride membrane (Merck Millipore, Billerica, MA, USA). The membranes were probed with primary rabbit antibodies as follows: β-actin (1:1,000, Rabbit, ab8227, Abcam, Cambridge, UK), EZH2 (# 5246, 1:1,000, Rabbit, CST, USA), phosphorylated-STAT3 (p-STAT3) (1:2,000, Rabbit, ab76315, Abcam), STAT3 (1:1,000, Rabbit, ab68153, Abcam), cleaved-caspase3 (#9661, 1:1,000, Rabbit, CST), and cleaved-poly ADP-ribose polymerase (cleaved-PARP) (#5625, 1:1,000, Rabbit, CST). The results were visualized using horseradish peroxidase-conjugated goat anti-rabbit immunoglobulin G (IgG) (ab205718, 1:2,000, Abcam) and enhanced chemiluminescence detection reagents. Image J software was used to analyze relative protein expression by analyzing the ratio of intensity of protein bands to be tested against that of β-actin.

### Reactive Oxygen Species (ROS) and Malondialdehyde (MDA) Measurement

ROS Assay Kit and Lipid Peroxidation MDA Assay Kit (Beyotime Institute of Biotechnology, Shanghai, China) were used for assays to detect levels of ROS and MDA, respectively.

### Cell Counting Kit-8 (CCK-8) Assay

HUVECs in the logarithmic growth phase were detached using 0.25% trypsin to form a single-cell suspension, of which 100 μl was seeded into 96-well-plates at a concentration of 5 × 10^4^ cells/ml. Three replicates were set in each group. Cells were incubated with 5% CO_2_ at 37°C for 24 and 48 h. At 1 h before the termination of culture, each well was added with 100 μl CCK-8 reagent (Beyotime). After further incubation for 1 h, the parameters of the enzyme label instrument (BD Biosciences, Franklin Lakes, NJ, USA) were set and the absorbance value of each well was measured at 450 nm.

### Cell Apoptosis Assays

Cell suspension (5 × 10^5^ cells, 0.5 ml) was transferred from the cell culture plate to a clean centrifuge tube, followed by incubation with staining solution and resuspension with a precooled 1× binding buffer (0.5 ml). Cells were incubated with 5 μl Annexin V-fluorescein isothiocyante (Beyotime) and 10 μl propidium iodide (Beyotime) without light exposure for 15 min. Finally, a flow cytometer (BD Biosciences, NJ, USA) was utilized to detect apoptosis.

### Dual Luciferase Reporter Gene Assay

A dual luciferase reporter gene assay was performed to identify whether EZH2 was a direct target gene of miR-200a. EZH2 3′-untranslated region (3′-UTR) gene fragments were artificially synthesized and introduced into pMIR-reporter (Promega, Madison, WI, USA) using endonuclease sites *SpeI* and *Hind III*. Mutation sites (MUT) of complementary sequences of seed sequences were designed on EZH2 wild-type (WT) plasmids. After restriction endonuclease digestion, the target fragment was inserted into the pMIR-reporter plasmid using T4 DNA ligase. The verified WT and MUT of EZH2 were cotransfected with miR-200a mimic and NC-mimic into HEK293 cells (Shanghai Beinuo Biotechnology Co., Ltd., Beijing, China). The cells were collected and split after transfection for 48 h. The Dual Luciferase Reporter Assay System kit (Promega) was used to detect the activity on the Glomax20/20 luminometer (Promega). Luciferase activity = firefly luciferase/renilla luciferase.

### Chromatin Immunoprecipitation (ChIP) Assay

The EZ-Magna ChIP reagent kit (EMD Millipore, MA, USA) was used for conducting the ChIP assay. HUVECs were fixed with 4% paraformaldehyde according to the manufacturer's instructions. The samples were incubated with glycine for 10 min to produce DNA–protein crosslink. Subsequently, the cells were lysed with a cell lysis buffer and a nuclear lysis buffer and treated with ultrasound to produce 200–300 BP chromatin fragments. Magnetic protein A beads with antibodies were used to precipitate lysate. The NC group was added with rabbit antibody to IgG (ab171870, Abcam), and an anti-EZH2 group was added with EZH2 antibody (#5246, 1:100, Rabbit, CST). Thereafter, RT-qPCR was performed to analyze the precipitated DNA and to quantify the promoter sequence of STAT3.

### Immunoprecipitation (IP) Assay

HUVECs treated with si-NC and siRNA targeting EZH2 were incubated for 48 to conduct the IP assay. Cells were collected and lysed using a lysis buffer supplemented with protease inhibitors, incubated on ice for 15 min, and cleared by centrifugation at 13,200 rpm at 4°C for 15 min. Total protein lysate (500 mg) was subjected to IP with the EZH2 (#5246, CST), STAT3 (#9139, CST), and methylated lysine (ab174719, Abcam) at 4°C overnight. Samples were then subjected to Western blot analysis.

### Enzyme-Linked Immunosorbent Assay (ELISA)

Whole blood was collected and centrifuged at 3,000 rpm for 30 min at room temperature to separate the serum. The concentration of tumor necrosis factor-α (TNF-α), interleukin-1β (IL-1β), and IL-6 in the culture supernatant was determined by mouse TNF-α ELISA kit (ab208348), mouse IL-1β ELISA kit (ab100704), and mouse IL-6 ELISA kit (ab100712), respectively. The absorbance of each well was determined at the wavelength of 450 nm using a microplate reader (BioTek, VT, USA), and analyzed by Origin 9.5 software. Moreover, the concentration of TNF-α, IL-1β, IL-6, and HMGB1 in HUVECs was determined by human TNF-α ELISA kit (ab181421), human IL-1β ELISA kit (ab46052), human IL-6 ELISA kit (ab178013), and human HMBG1 ELISA kit (ab77302), respectively.

### Histological Analyses

Hematoxylin and eosin (HE) staining: The aortas of the experimental mice were isolated, fixed with 4% paraformaldehyde, and embedded in paraffin. After dewaxing and hydration, the sections were treated with HE staining. Pathological changes in blood vessels were observed under a Leica microscope (Leica M205C).

#### Oil Red O Staining

In order to observe the degree of aortic root lesions, the cross sections of the aortic roots (10 μm) in each group of mice were stained with 0.5% oil-red-O staining (Sigma-Aldrich Chemical Company, St. Louis, MO, USA) for 30 min and then with hematoxylin (Servicebio, Wuhan, China) for 20 s. Representative images of lesions were captured by a Leica microscope (Leica M205C) and analyzed using Image-Pro Plus software (19).

#### Immunohistochemistry

The paraffin-embedded sections were treated with immunohistochemical staining using the primary antibody EZH2 (#5246, 1:50, Rabbit, CST), HMGB1 (1:250, Rabbit, ab79823, Abcam), p-STAT3 (1:500, Rabbit, ab76315, Abcam), cleaved-caspase3 (#9661, 1:200, Rabbit, CST), and cleaved-PARP (#5625, 1:150, Rabbit, CST). The samples were observed under a Leica microscope (Leica M205C). Positive stains were scored according to a previously published method (20).

### Statistical Analysis

All data were summarized as mean ± standard deviation of values from at least three independent experiments conducted in triplicate. Unpaired *t*-test was used to compare data from two groups and one-way analysis of variance (ANOVA) to compare data from multiple groups. A value of *p* < 0.05 indicated statistical significance. All analyses were performed using the SPSS 21.0 software (IBM Corp. Armonk, NY, USA).

## Results

### Expression Pattern of miR-200a in ox-LD-Induced HUVECs

To investigate the roles of miR-200a in atherosclerosis, RT-qPCR was used to measure the miR-200a expression in ox-LD-induced HUVECs and showed that ox-LDL inhibited miR-200a expression in a dose-dependent and time-dependent manner (*p* < 0.05; Figure 1), suggesting that miR-200a may be associated with the development of atherosclerosis.

**Figure 1:** miR-200a is downregulated in ox-LDL-induced HUVECs. **(A)** miR-200a expression in HUVECs treated with 0, 20, and 40 μg/ml ox-LDL at 24 h determined using RT-qPCR, normalized to U6. **(B)** miR-200a expression in HUVECs treated with 20 μg/ml ox-LDL at 0, 24, and 48 h determined using RT-qPCR, normalized to U6. *(relative to untreated HUVECs) indicates *p* < 0.05 by one-way ANOVA/Tukey's *post-hoc* test.

### miRNA-200a Protected HUVECs Against ox-LDL-Induced Apoptosis and Inflammation

HUVECs were treated with exogenous miR-200a mimic to further explore the effects of miR-200a on ox-LDL-induced HUVECs. RT-qPCR displayed that miR-200a expression increased in ox-LDL-induced HUVECs treated with exogenous miR-200a mimic (*p* < 0.05; Figure 2A). ROS and MDA are important indices to evaluate HUVEC injury caused by atherosclerosis. The levels of ROS and MDA increased in HUVECs treated with ox-LDL and decreased after restoration of miR-200 in the presence of ox-LDL (*p* < 0.05; Figures 2B,C). CCK-8 assay and flow cytometry revealed that ox-LDL inhibited cell viability and induced apoptosis, whereas opposing results were noted in ox-LDL-induced HUVECs treated with exogenous miR-200a mimic (*p* < 0.05; Figures 2D,E). Moreover, Western blot analysis and ELISA presented that ox-LDL elevated levels of cleaved-caspase3 and cleaved-PARP, TNF-α, IL-1β, and IL-6 in the culture supernatant of ox-LDL-induced HUVECs, whereas these levels were significantly lowered in HUVECs treated with exogenous miR-200a mimic (*p* < 0.05; Figures 2F–I). These results together suggested that miR-200a could inhibit cell injury, apoptosis, and inflammation of ox-LDL-induced HUVECs.

**Figure 2:** MiRNA-200a protects HUVECs against ox-LDL-induced apoptosis and inflammation. HUVECs were cultured with ox-LDL or treated with exogenous miR-200a mimic (with NC mimic as control). **(A)** miR-200a expression level in HUVECs determined using RT-qPCR, normalized to U6. **(B)** ROS level in HUVECs measured with ROS Assay Kit. **(C)** MDA level in HUVECs measured with ROS Assay Kit. **(D)** Cell viability of HUVECs detected by CCK-8 assay. **(E)** Apoptosis of HUVECs detected by flow cytometry. **(F)** Protein levels of cleaved-caspase3 and cleaved-PARP in HUVECs determined by Western blot analysis, normalized to β-actin. **(G–I)** Concentration of TNF-α, IL-1β, and IL-6 in the culture supernatants of HUVECs measured by ELISA. *(relative to untreated HUVECs) and ^#^(relative to ox-LDL-treated HUVECs) indicate *p* < 0.05 by one-way ANOVA/Tukey's *post-hoc* test.

### miR-200a Targeted and Downregulated EZH2 in HUVECs

In order to further study, the downstream mechanisms of miR-200a, a web-based bioinformatic resource TransmiR was used and it was predicted that miR-200a interacted with 72 transcription regulators (Figure 3A). Using StarBase and miRTarBase databases, it was predicted that the target genes had binding sites for miR-200a. Venn online tool was used to identify the overlap in prediction results obtained from TransmiR, StarBase, and miRTarBase, and suggested that miR-200a could bind to four genes (ZEB1, Smad3, EZH2, and ZEB2; Figure 3B). Using StarBase, it was predicted that miR-200a could target EZH2 (Figure 3C). A dual luciferase reporter gene assay showed that the luciferase activity of WT-EZH2 3′-UTR was significantly inhibited by miR-200a (*p* < 0.05), but no difference was found in MUT-EZH2 3′-UTR (*p* > 0.05; Figure 3D). A dual luciferase reporter gene assay was used to further verify that miR-200a targeted EZH2 in mice in order to analyze the functional mechanism of miR-200a targeting EZH2 in mice *in vivo*. The findings indicated that luciferase activity of miR-200a/WT-EZH2 was significantly decreased (*p* < 0.05), but no difference was found in MUT-EZH2 3′-UTR (*p* > 0.05; Figure 3E), suggesting that miR-200a could specifically bind to EZH2. In HUVECs, mRNA and protein level was significantly reduced in HUVECs treated with exogenous miR-200a mimic (*p* < 0.05; Figures 3F,G). Moreover, RT-qPCR and Western blot analysis showed that ox-LDL promoted EZH2 expression in a dose-dependent and time-dependent manner (*p* < 0.05; Figures 3H–J). Therefore, the obtained data suggested that miR-200a could target EZH2 and inhibit EZH2 expression.

**Figure 3:** miR-200a targets EZH2 and downregulates EZH2 in HUVECs. **(A)** The interacting transcription factors that interacted with miR-200a predicted using TransmiR database (http://www.cuilab.cn/transmir). **(B)** Venn graph (http://bioinformatics.psb.ugent.be/webtools/Venn/) of intersection of prediction results of TransmiR with StarBase database (http://starbase.sysu.edu.cn/) and miRTarase database (http://mirtarbase.mbc.nctu.edu.tw/php/index.php). **(C)** Binding site of miR-200a EZH2 3′-UTR. **(D)** Target relationship between miR-200a and EZH2 in HUVECs detected using dual-luciferase reporter gene assay. **(E)** Target relationship between miR-200a and EZH2 in arterial tissues of ApoE^−/−^ mice detected using dual-luciferase reporter gene assay. HUVECs were treated with exogenous miR-200a mimic (with NC mimic as control). **(F)** EZH2 mRNA level in HUVECs determined by RT-qPCR, normalized to GAPDH. **(G)** EZH2 protein level in HUVECs determined by Western blot analysis, normalized to β-actin. HUVECs were treated with 0, 20, and 40 μg/ml ox-LDL for 24 h. **(H)** EZH2 mRNA level in HUVECs determined by RT-qPCR. HUVECs were treated with 0, 20, and 40 μg/ml ox-LDL for 24 h. **(I)** EZH2 mRNA level in HUVECs treated with 20 μg/ml ox-LDL for 0, 24, and 48 h determined by RT-qPCR. **(J)** EZH2 protein level in HUVECs determined by Western blot analysis, normalized to β-actin. HUVECs were treated with 0, 20, and 40 μg/ml ox-LDL for 24 h as well as treated with 20 μg/ml ox-LDL for 0, 24, and 48 h.*indicates *p* < 0.05 compared with untreated HUVECs or empty vector-treated HUVECs. Unpaired *t*-test was used to compare data from two groups and one-way ANOVA/Tukey's *post-hoc* test to compare data from multiple groups.

### Silencing of EZH2 Mimicked the Protective Effects of miR-200a on HUVECs Against ox-LDL-Induced Injury

Next, HUVECs were treated with siRNA targeting EZH2-1 and EZH2-2 to verify whether miR-200a affected cell injury, apoptosis, and inflammation in ox-LDL-induced HUVECs via regulation of EZH2. RT-qPCR results displayed that EZH2 expression decreased in HUVECs treated with siRNA targeting EZH2-1 or EZH2-2 (*p* < 0.05; Figure 4A), and thus, the HUVECs treated with siRNA targeting EZH2-1 were selected for further experiments. RT-qPCR and Western blot analysis indicated that EZH2 expression was elevated in HUVECs treated with exogenous miR-200a mimic and expression vectors containing EZH2 (*p* < 0.05; Figures 4B,C). The levels of ROS and MDA were decreased in HUVECs treated with siRNA targeting EZH2, and they were increased in HUVECs treated with exogenous miR-200a mimic and expression vectors containing EZH2 (*p* < 0.05; Figures 4D,E). Flow cytometry and CCK-8 assays revealed that apoptosis was inhibited and cell viability was promoted in HUVECs treated with siRNA targeting EZH2, whereas the results were opposite in HUVECs treated with exogenous miR-200a mimic and expression vectors containing EZH2 (*p* < 0.05; Figures 4F,H). In addition, Western blot analysis and ELISA showed that the levels of cleaved-caspase3 and cleaved-PARP, TNF-α, IL-1β, and IL-6 were reduced in the culture supernatant of HUVECs treated with siRNA targeting EZH2, while these levels were elevated in HUVECs treated with exogenous miR-200a mimic and expression vectors containing EZH2 (*p* < 0.05; Figures 4G,I–K). Together, these data demonstrated that miR-200a contributed to the suppression of cell injury, apoptosis, and inflammation of ox-LDL-induced HUVECs by inhibiting EZH2.

**Figure 4:** Silencing of EZH2 enables protective effects on HUVECs against ox-LDL-induced injury similar to miRNA-200a upregulation. HUVECs were treated with siRNA targeting EZH2-1 and EZH2-2 (with si-NC as control). **(A)** Interference efficiency of EZH2 in HUVECs measured by RT-qPCR. HUVECs were treated with siRNA targeting EZH2 (with si-NC as control) and exogenous miR-200a mimic and expression vectors containing EZH2 (with miR-200a mimic + oe-NC as control). **(B)** EZH2 expression in HUVECs determined using RT-qPCR, normalized to GAPDH. **(C)** EZH2 expression in HUVECs determined using Western blot analysis, normalized to β-actin. **(D)** ROS level in HUVECs measured with the ROS Assay Kit. **(E)** MDA level in HUVECs measured with the ROS Assay Kit. **(F)** Apoptosis of HUVECs detected by flow cytometry. **(G)** Protein levels of cleaved-caspase3 and cleaved-PARP in HUVECs determined by Western blot analysis, normalized to β-actin. **(H)** Cell viability of HUVECs detected by CCK-8 assay. **(I–K)** Concentration of TNF-α, IL-1β, and IL-6 in the culture supernatant of HUVECs measured by ELISA. *(relative to scramble siRNA-treated HUVECs) and ^#^(relative to miR-200a-mimic + oe–NC) indicate *p* < 0.05 by one-way ANOVA/Tukey's *post-hoc* test.

### EZH2 Methylated STAT3 and Activated p-STAT3/HMGB1 Activity in ox-LD-Induced HUVECs

The web-based bioinformatics resource “hTFtarget” was used, and it was predicted that EZH2 can target STAT3 (Figure 5A). Western blot analysis showed that ox-LDL induced expression of STAT3 and p-STAT3 in a dose- and time-dependent manner (*p* < 0.05; Figure 5B). IP assay was performed to detect the interaction between EZH2 and STAT3 in HUVECs (Figure 5C). ChIP assay revealed that EZH2 was enriched in the STAT3 promoter region in HUVECs treated with siRNA targeting EZH2 (*p* < 0.05; Figure 5D). IP assay showed that STAT3 methylation was inhibited in HUVECs treated with siRNA targeting EZH2 (*p* < 0.05; Figure 5E). Western blot analysis and ELISA displayed that the expression of p-STAT3 and HMGB1 decreased in HUVECs treated with siRNA targeting EZH2 (*p* < 0.05; Figure 5F). ELISA exhibited that ox-LDL promoted the HMGB1 level in a dose- and time-dependent manner (*p* < 0.05; Figures 5G,H). These findings confirmed that EZH2 methylated STAT3 and enhanced STAT3 activity by increasing tyrosine phosphorylation of STAT3, thereby leading to increased HMGB1.

**Figure 5:** EZH2 methylates STAT3 and activates p-STAT3/HMGB1 in ox-LDL-induced HUVECs. **(A)** EZH2 could target STAT3 predicted using the web-based bioinformatics resource hTFtarget (http://bioinfo.life.hust.edu.cn/hTFtarget#!/). HUVECs were treated with 0, 20, and 40 μg/ml ox-LDL. **(B)** Protein levels of p-STAT3/STAT3 in HUVECs at 0, 24, and 48 h measured using Western blot analysis, normalized to β-actin. HUVECs were treated with siRNA targeting EZH2. **(C)** The interaction between EZH2 and STAT3 in HUVECs detected by IP assay. **(D)** Enrichment of EZH2 in the STAT3 promoter region in HUVECs detected by ChIP assay. **(E)** Effect of EZH2 on STAT3 methylation in HUVECs detected by IP assay. **(F)** Protein levels of p-STAT3/STAT3 in HUVECs measured using Western blot analysis, normalized to β-actin, and HMGB1 concentration determined by ELISA. **(G)** HMGB1 concentration at 24 h in HUVECs determined using ELISA. HUVECs were treated with 0, 20, and 40 μg/ml ox-LDL for 24 h. **(H)** HMGB1 concentration in HUVECs determined using ELISA. HUVECs were treated with 20 μg/ml ox-LDL for 0, 24, and 48 h. *(relative to IgG or untreated HUVECs) and ^#^(relative to scramble siRNA-treated HUVECs) indicate *p* < 0.05 by one-way ANOVA/Tukey's *post-hoc* test.

### EZH2-Mediated Methylation of STAT3 Enhanced ox-LDL-Induced Injury on HUVECs by Activating p-STAT3/HMGB1

HUVECs were treated with siRNA targeting HMGB1 or siRNA targeting EZH2 and expression vectors containing HMGB1 to further verify the function of EZH2 activating p-STAT3-HMGB1 in HUVECs in the following experiments. RT-qPCR exhibited that HMGB1 expression decreased in HUVECs treated with siRNA targeting HMGB1-1 or HMGB1-2 (*p* < 0.05; Figure 6A), and the HUVECs treated with siRNA targeting HMGB1-1 were selected for further experiments. Western blot analysis demonstrated that the expression of p-STAT3 and HMGB1 was elevated in HUVECs treated with siRNA targeting EZH2 and expression vectors containing HMGB1 (*p* < 0.05; Figure 6B). The levels of ROS and MDA were decreased in HUVECs treated with siRNA targeting HMGB1 and increased in HUVECs treated with siRNA targeting EZH2 and expression vectors containing HMGB1 (*p* < 0.05; Figures 6C,D). CCK-8 assay and flow cytometry revealed that cell viability was enhanced and apoptosis was inhibited in HUVECs treated with siRNA targeting HMGB1, while the opposite results were observed in HUVECs treated with siRNA targeting EZH2 and expression vectors containing HMGB1 (*p* < 0.05; Figures 6E,F). Furthermore, Western blot analysis and ELISA revealed that levels of cleaved-caspase3 and cleaved-PARP, TNF-α, IL-1β, and IL-6 were reduced in the culture supernatants of HUVECs treated with siRNA targeting HMGB1, whereas these levels were elevated in HUVECs treated with siRNA targeting EZH2 and expression vectors containing HMGB1 (*p* < 0.05; Figures 6G–J). Taken together, these results indicated that EZH2 induced apoptosis and inflammation of ox-LDL-induced HUVECs via the activation of p-STAT3-HMGB1.

**Figure 6:** EZH2-mediated methylation of STAT3 enhances ox-LDL-induced injury in HUVECs by activating p-STAT3/HMGB1. **(A)** Interference efficiency of HMGB1 in HUVECs measured by ELISA. HUVECs were treated with siRNA targeting HMGB1 (with si-NC as control) or siRNA targeting EZH2 and expression vectors containing HMGB1 (with si- EZH2 + oe-NC as control). **(B)** Protein levels of p-STAT3/STAT3 in HUVECs determined using Western blot analysis, normalized to β-actin, and HMGB1 level determined by ELISA. **(C)** ROS levels in HUVECs measured with the ROS Assay Kit. **(D)** MDA levels in HUVECs measured with the ROS Assay Kit. **(E)** Cell viability of HUVECs detected by CCK-8 assay. **(F)** Apoptosis of HUVECs detected by flow cytometry. **(G)** Protein levels of cleaved-caspase3 and cleaved-PARP in HUVECs determined by Western blot analysis, normalized to β-actin. **(H–J)** Concentration of TNF-α, IL-1β, and IL-6 in the culture supernatant of HUVECs measured by ELISA. *(relative to scramble siRNA-treated HUVECs) and ^#^(relative to siRNA-targeting EZH2-treated HUVECs) indicate *p* < 0.05 by one-way ANOVA/Tukey's *post-hoc* test.

### The Anti-atherosclerotic Role of miR-200a in Atherosclerotic Mice *in vivo*

ApoE^−/−^ mice were fed with a high-fat diet and injected with miR-200a agomir to further explore the mechanisms by which miR-200a inhibiting p-STAT3-HMGB1 may participate in atherosclerosis by repressing EZH2 expression. RT-qPCR (Figure 7A) demonstrated that miR-200a expression was decreased in ApoE^−/−^ mice fed with a high-fat diet. Injection of miR-200a agomir increased the expression of miR-200a in arterial tissues of the mice fed with a high-fat diet (*p* < 0.05). HE and oil red O staining revealed that atherosclerosis mouse models were successfully established, showing increased size and lipid content of the lesions, while upregulated miR-200a alleviated atherosclerosis by inhibiting lipid content (*p* < 0.05; Figures 7B–E). ELISA and immunohistochemical staining exhibited that the levels of TNF-α, IL-1β, IL-6, EZH2, p-STAT3, HMGB1, cleaved-caspase3, and cleaved-PARP were elevated in arterial tissues of mice fed with a high-fat diet, while these levels reduced in arterial tissues of mice fed with a high-fat diet and injected with miR-200a agomir (*p* < 0.05; Figures 7F–I). Thus, it can be concluded that miR-200a suppressed the progression of atherosclerosis by inhibiting EZH2 and p-STAT3-HMGB1 *in vivo*.

**Figure 7:** The antiatherosclerotic role of miR-200a in atherosclerotic mice. ApoE^−/−^ mice were fed with a high-fat diet (with ND + NC as control) and injected with miR-200a agomir (with HFD + NC as control). **(A)** miR-200a expression (normalized to U6) in arterial tissues of ApoE^−/−^ mice (*n* = 10) determined using RT-qPCR. **(B)** Oil red O staining images of arterial tissues of ApoE^−/−^ mice. **(C)** Total aortic lesions detected by oil red O staining. **(D)** Lipid deposition of arterial tissues of ApoE^−/−^ mice detected by oil red O staining (×100), red indicating lipid-rich plaque. **(E)** Atherosclerotic lesions in arterial tissues of ApoE^−/−^ mice detected by HE staining (×100; × 400). **(F–H)** Concentration of TNF-α, IL-1β, and IL-6 in the serum of ApoE^−/−^ mice measured by ELISA. **(I)** Expression levels of EZH2, p-STAT3, STAT3, HMGB1, cleaved-caspase3, and cleaved-PARP in the arterial tissues of ApoE^−/−^ mice measured by immunohistochemical staining (×400). *(relative to normal diet-treated mice) and ^#^(relative to high-fat diet-treated mice) indicate *p* < 0.05 by one-way ANOVA/Tukey's *post-hoc* test.

## Discussion

As a persistent inflammatory vascular disorder, atherosclerosis remains a major cause of death and disability globally (6). In recent years, multiple miRNAs have been reported to play functional roles in the prevention of endothelial inflammatory response and atherosclerotic lesion formation, thereby providing a protective effect against atherosclerosis (21). In the present study, atherosclerosis mouse models were established with an aim to explore the effects of miR-200a on the viability, apoptosis, cell injury, and inflammation of HUVECs. Taken together, our findings provided evidence that the upregulation of miR-200a repressed the activation of the STAT3/HMGB1 axis by inhibiting EZH2 expression, thus suppressing cell injury, apoptosis, and inflammation while promoting viability of ox-LDL-induced HUVECs, which helped alleviate atherosclerosis progression.

Our early results implied that miR-200a was downregulated in ox-LDL-induced HUVECs, and the upregulation of miR-200a could promote cell viability and inhibit cell injury, apoptosis, and inflammation of ox-LDL-induced HUVECs so as to suppress the progression of atherosclerosis. It is known that atherosclerosis is accompanied by the release of inflammatory cytokines, such as IL-1β and IL-18, which can be triggered by inflammasomes (5). ox-LDL can induce ROS secretion, inflammatory responses, and apoptosis of endothelial cells for atherosclerosis (22). The dysregulation of miRNAs exerts effects on the development and progression of atherosclerosis (23). Tang and Yang (24) have revealed that miR-126 was poorly expressed in ox-LDL-treated HUVECs, and restoration of miR-126 attenuates ox-LDL-induced HUVEC injury by inhibiting apoptosis. MiR-200a expression is reported to be reduced in multiple tumors (9). Lo et al., found that miR-200a exerts effects on the human aortic endothelial cells (10). The MiR-200 family is considered to facilitate improved β-cell function by maintaining the balance between differentiation and proliferation during metabolic diseases including atherosclerosis (25). Another recent study has demonstrated that miR-126-5p enhances endothelial cell proliferation to suppress atherosclerosis progression (26). These and similar experimental evidences support the notion that miR-200a might bear potential as a valuable therapeutic target for reversal of atherosclerosis.

In the present study, bioinformatics analysis and dual luciferase reporter gene assay together demonstrated that miR-200a could target EZH2 and suppress EZH2 expression. It has been reported earlier that miR-200a expression is negatively correlated with EZH2 expression (27). Emerging evidence has exhibited that EZH2 can be potentially targeted by miRNAs, and that EZH2 overexpression can promote the progression of atherosclerosis in ApoE^−/−^ mice fed with a high-fat diet (12). EZH2 is upregulated in ApoE^−/−^ mice affected with atherosclerosis, and contributes to the accumulation of lipids and formation of foam cells to aggravate the progression of atherosclerosis (28), which suggests that a downregulation of EZH2 could relieve atherosclerosis. These findings present a rationale to investigate if a depletion of EZH2 underlies the anti-atherosclerotic effect of miR-200a.

The present study also confirmed that EZH2 could activate p-STAT3-HMGB1 by promoting STAT3 methylation. EZH2 can bind to and methylate STAT3 to enhance the STAT3 activity via elevation of STAT3 phosphorylation (14). Luo et al. (29) have demonstrated that a switch in EZH2 function from histone-methyltransferase to non-histone methyltransferase led to methylation of STAT3 and promoted prostate cancer neuroendocrine differentiation. STAT3 also serves as a regulator of HMGB1 expression in human lung microvascular endothelial cells and thereby affects inflammatory responses (16). The current study has found that miR-200a inhibited cell injury, apoptosis, and inflammation of ox-LDL-induced HUVECs by suppressing EZH2 and p-STAT3-HMGB1, thereby repressing the progression of atherosclerosis. Upregulation of another miRNA, miR-181b, is also reported to attenuate the progression of atherosclerosis by inhibiting STAT3, which eventually leads to repressed cell growth, cell cycle arrest, and apoptosis (15). In another instance, elevated miR-126 is shown to inhibit inflammation and ROS production in endothelial cells by suppressing HMGB1 expression in the diabetic vascular endothelium (30). HMGB1 is also confirmed to participate in atherosclerosis development and is targeted by miR-328 such that miR-328 overexpression inhibits inflammation, oxidative stress, and apoptosis of ox-LDL-treated HUVECs (7). Combining insights obtained from previous studies with our results, a regulatory network involved in antagonizing atherosclerosis progression may be proposed, where miR-200a restoration inhibits EZH2 expression to disrupt the STAT3/HMGB1 axis.

The findings of the study need to be viewed in light of its limitations. Endothelial cells play an important role in the pathogenesis of inflammation, transplant rejection, and tumor metastasis. Thus, HUVECs have been used in research focused on endothelial cells. However, in recent years, human saphenous vein endothelial cells (HSVECs) have emerged as a better *in vitro* alternative as compared to HUVECs from a perspective of pathology. HSVECs have been found to be more sensitive with ox-LDL and less responsive to cytokines, which may be attributed to the expression of adhesion molecules as well as the adhesion and transportation of leukocytes (31). Thus, the current findings should be validated in alternative cell models such as HSVECs. In addition to the reported regulatory role of ox-LDL in HUVECs reported in our study, ox-LDL has been noted to impair angiogenesis by inhibiting vascular endothelial growth factor receptor 2 expression (32), suggesting that further research is essential for a complete understanding of its roles. Importantly, miR-200a may mediate atherosclerosis progression depending on other pathways besides immunomodulation discussed in our study. For instance, miR-200a has been demonstrated to facilitate inflammation in vascular smooth muscle cells (33), suggesting that pro-inflammatory action of miR-200a may be dependent on smooth muscle cells. Also, miR-200a has been elucidated to promote apoptosis (34). Notably, apoptosis of vascular smooth muscle cells is one of the distinctive features of atherosclerosis (35). Hereby, the regulatory role of miR-200a in the context of atherosclerosis requires further investigation.

## Conclusions

In conclusion, our study demonstrated that upregulation of miR-200a could inhibit the expression of EZH2, which potentially suppressed the development of atherosclerosis through inactivation of the STAT3/HMGB1 axis (Figure 8). Our study also provided further insights into the regulatory network and the underlying roles of miR-200a-mediated regulation of EZH2 via the STAT3/HMGB1 axis in atherosclerosis. However, further investigations are required to evaluate its potential application in preclinical models and clinical trials in patients with atherosclerosis. Additional studies are essential in order to adequately define and clarify the detailed mechanisms by which miR-200a interacts with EZH2 and the STAT3/HMGB1 axis to influence atherosclerosis progression.

**Figure 8:** Schematic representation of the regulatory mechanism of miR-200a involvement in atherosclerosis. Overexpression of miR-200a inhibits EZH2 and HMGB1 expression by suppressing methylation and activation of STAT3 to inhibit cell injury, apoptosis, and inflammatory response, thereby repressing the progression of atherosclerosis.

## Data Availability Statement

The raw data supporting the conclusions of this article will be made available by the authors, without undue reservation, to any qualified researcher.

## Ethics Statement

All animal experiments were approved by the Ethics Committee of Medical Experiment Animals in the College of Basic Medicine of Jilin University.

## Author Contributions

JW and PL wrote the paper and conceived and designed the experiments. BZ collected and provided the sample for this study. XX and JZ edited and revised the paper. All authors have read and approved the final submitted manuscript.

## Conflict of Interest

The authors declare that the research was conducted in the absence of any commercial or financial relationships that could be construed as a potential conflict of interest.
